# Evaluation of landscape created by erosion control dam using physiological and psychological indicators

**DOI:** 10.1371/journal.pone.0309804

**Published:** 2024-10-03

**Authors:** Yong-Rae Kim, Beom-Su Kim, Choyun Kim, Sang In Lee, Won-Shin Cho, Hyeongkeun Kweon, Chorong Song, Jung Il Seo

**Affiliations:** 1 Institute of Ecological Restoration, College of Industrial Sciences, Kongju National University, Yesan-gun, Chungcheongnam-do, Republic of Korea; 2 Department of Forest Science, College of Industrial Sciences, Kongju National University, Yesan-gun, Chungcheongnam-do, Republic of Korea; 3 Department of Crops and Forestry, Korea National University of Agriculture and Fisheries, Jeonju-si, Jeollabuk-do, Republic of Korea; Universita degli Studi di Pisa, ITALY

## Abstract

This study demonstrated the effect of differences in the exterior of erosion control dams (ECDs) on humans. We recruited 34 university students. Participants sat 1.4 m away from the display while wearing a device for measuring heart rate (HR) and heart rate variability. They (i) took a rest while viewing a gray screen for one minute; (ii) viewed a randomly displayed image of one of the three ECDs’ images for one minute; (iii) filled out questionnaires (using the semantic differential method and a profile of mood states) for five minutes; and (iv) took a rest to wash out residual sensitivity for five minutes. The process was repeated three times with three different ECD images. No significant difference was found between the participants’ HRs measured before and while viewing the images of the three ECDs with different exterior materials, although the HRs were significantly reduced when viewing the wood-attached ECD compared with the concrete-exposed ECD. Participants perceived the concrete-exposed and stone-attached ECDs artificially, while they felt the wood-attached ECD naturally. In addition, the vigor score was significantly increased while total mood disturbance was significantly decreased when viewing the wood-attached ECD. However, there were no significant differences in other indicators, and participants’ responses to the exteriors of the ECDs were positive overall. Our findings show that people do not physiologically and psychologically perceive ECDs negatively. Therefore, securing stability against sedimentary disasters should be a priority before using the landscape elements of an ECD.

## Introduction

Approximately 62.6% of the land area in the Republic of Korea is covered with steep and undulating mountainous forests [1], the population density is the 27th in the world [2], and thus, infrastructure such as public institutions, houses, and factories are adjacent to forests [3–5]. Developmental activities in Korea are frequent in the mountainous forests around the urban environments due to the expansion of the living area accompanied by the urban concentration of the population [6, 7], so the physical separation distance between forests and people is small. Under these conditions, geomorphic disturbances such as landslides and debris flows can lead to enormous human and property damage. A typical example is the Mt. Umyeon landslide that occurred in Seoul, Korea in 2011. This landslide killed a total of 16 people and damaged approximately USD 16 million worth of property [8, 9].

The Korea Forest Service and local governments have been installing erosion control dams (ECDs) over three decades to prevent the damage caused by such sedimentary disasters and to preserve ultimately forest ecosystems [1]. An ECD is a representative cross-sectional structure that protects the downstream area from geomorphic disturbances such as landslides and debris flows by reducing the water flow velocity as well as controlling sediment discharge [10, 11], and is also called check dam or sabo dam [12, 13]. It is constructed mainly of concrete to secure sufficient strength above the standard level against impacts caused by landslides and debris flows [14, 15]. However, some environmental movement groups and media in Korea point out that despite the disaster reduction effect of ECDs, the appearance (i.e., surface material) of ECDs does not harmonize with nature, damaging the forest landscape [16].

Accordingly, the Korea Forest Service is implementing a policy to encourage the application of techniques that give ECDs a nature-positive appearance so that there is no sense of separation from the surrounding forests, in addition to greening the area inevitably damaged by being used as a workspace for heavy equipment [17]. Typical examples include attaching stones or embalmed wood on the surface of a concrete dam. For such government level efforts to lead to a meaningful ending, objective evaluation techniques for the landscape created by an ECD must be prepared, and the evaluation results should feed back to the design of the ECD. However, while the physical stability of ECDs against sedimentary disasters has been evaluated worldwide, little evaluation has been made of its effect on the landscape. As an exception, Lee et al. [18] conducted an on-site self-written survey to identify preferences from a landscape point of view by providing respondents with photos of ECDs finished with stones (a nature-positive material) or concrete (a nature-negative material) and reported that ECDs finished with stones had a higher preference than those finished with concrete. Their survey technique has the advantage of intuitively reflecting respondents’ opinions. However, the images used in the survey have limitations, as it is difficult to directly and definitively compare the effects of the finishing materials of ECDs because the surrounding conditions, such as stream water discharge and vegetation cover, are not controlled.

Previous studies conducted in the fields of architecture and landscape mainly employed a method using sample materials (e.g., photo, brick) obtained from indoor or outdoor as stimuli for subjects in specific spaces and writing their perceptions and preferences in questionnaires [e.g., 19–23]. For instance, Wastiels et al. [19] explored the possibilities relating material experience in architecture to technical material parameters and uses the perceived warmth of indoor wall materials. In their study, various building materials were assessed technically and, for each material sample, a separate questionnaire page was provided and participants completed a list of 15 attribute pairs based on a 9-point itemized rating scale. Abkar et al. [20] compared images displaying urban built landscape and urban natural landscapes to determine subjects’ visual preference for urban landscapes. In their study, participants assessed each of the 24 settings with 17 items including a target variable, preference and four predictors of preference (16 items), and all items in the questionnaire were rated on a 7-point Likert scale of agreement ranging from 1 (not at all) to 7 (a great deal). Burnard et al. [21] aimed to understand user perceptions of building material naturalness, and their objectives were achieved by conducting surveys asking users to rate the naturalness of building materials. The surveys were conducted in three countries to determine if regional or cultural traditions, especially related to building and material use, influence user perceptions of building material naturalness. However, these survey techniques have the disadvantage being able to provide inaccurate or dishonest answers because anonymity is guaranteed and immediate responsibility is not given in filling out the questionnaire, which can distort the survey results.

To overcome such limitations of survey techniques, studies using human physiological and psychological indicators, which have a somewhat high degree of control over experimental conditions, are being developed in various scientific fields [22–25]. Physiological indicators can obtain information on nonverbal or personal characteristics by measuring and analyzing variations in heart rate, blood oxygen saturation, and sympathetic and parasympathetic nerves systems [26]. Psychological indicators quantitatively identify changes in subjective perception according to given conditions by measuring and analyzing indicators of self-report questions expressing human emotions or moods [27, 28]. In the forest science field, several studies related to forest welfare and therapy have been conducted using physiological and psychological indicators. Park et al. [29] measured the effect of forest bathing on the physiological and psychological responses of the human body and reported that the degree of negative emotions felt by humans in forests significantly decreased compared with those in cities. Song et al. [30] also measured physiological and psychological reactions, including brain activity, when humans look at pictures of forests and cities via a display device and suggested that humans’ negative emotions decrease and comfortable and relaxed perceptions increase when looking at pictures of forests compared with cities. However, no study has dealt with the physiological and psychological effects of the landscape created by an ECD, a public facility for preventing damages caused by geomorphic disturbances such as landslides and debris flows in stream water zone.

Against this research background, this study aimed to reveal the physiological and psychological effects on the human body resulting from differences in an ECD’s exterior (finishing materials). Furthermore, guidelines for constructing ECDs while considering the natural landscape are presented based on the results. To this end, we measured heart rate (HR) and heart rate variability (HRV) to examine participants’ physiological responses while viewing images of three different exterior types (i.e., concrete-exposed, stone-attached, and wood-attached) of ECDs via a display device. We then identified a participant’s psychological state using the semantic differential (SD) method and a profile of mood state (POMS). We finally compared the differences in the results of the collected physiological and psychological indicators.

## Methods

### 1. Participants

A notice of participant recruitment was posted on the bulletin board of the College of Industrial Sciences, Kongju National University, from March 23 to 31, 2023.

The recruitment of participants was aimed at students at the College of Industrial Sciences, Kongju National University in their early 20s without any preconceived notions because they did not receive professional education in ECDs. However, those currently in treatment for any disease, those with a history of allergic reactions or multiple drug side effects, those with a history of heart disease, and those with visual abnormalities were excluded from the recruitment.

The sample size required for this experiment was calculated using G*Power software (University of Kiel, Kiel, Germany) [31]. From the calculation, a minimum of 28 participants were required to detect statistically significant differences in the two-tailed test with an effect size of 0.25, significance level of 0.05, and power of 0.80. However, Lee [32] suggests that, considering the dropouts that may occur during clinical trials, the sample size should include an additional 10 to 20% of the minimum sample size to secure the desired power. Therefore, in this study, a total of 34 participants (19 males and 15 females) were voluntarily recruited, including 28 samples calculated using the G*Power software and 6 samples with a 20% dropout rate (Table 1).

**Table 1:** Participant characteristics (*n* = 34).

	Age (year)	Height (cm)	Weight (kg)	Body mass index (kg/m^2^)
Total (n = 34)	20.5±1.6	169.2±9.2	67.6±16.2	23.5±4.9
Male (n = 19)	20.8±1.6	175.7±6.0	72.6±15.0	23.4±3.8
Female (n = 15)	20.1±1.5	161.0±5.0	61.3±15.9	23.7±6.1

*Note*: All values were expressed as means ± standard deviations.

The study was conducted per the guidelines of the Declaration of Helsinki. All experimental procedures were carried out with the approval of the Institutional Review Board of Kongju National University (KNU-IRB), Republic of Korea (no. KNU-IRB_2023–014), and the participants signed a consent form provided by the KNU-IRB before proceeding with the experiment. Pre-registration, which is the practice of registering the hypotheses, methods, and/or analyses of a scientific study before it is conducted, was not performed in this study.

### 2. Experimental design

The experiment was performed at the laboratory where elements (noise, light, wind, etc.) interfering with the participants’ stability were blocked. The laboratory temperature and humidity were maintained at 24°C and 50%, respectively.

Upon arrival at the laboratory, participants voluntarily filled out consent forms after briefing to the purpose and procedure of the experiment before starting the experiments. After attaching the instrument for measuring physiological parameters, the participants sat comfortably 1.4 m away from the display so that the viewing angles based on the center point of the display were approximately ±24° wide and ±14° high, respectively, (i) taking a rest while looking at a gray screen for one minute; (ii) viewing a randomly displayed image of one of the three ECDs’ images for one minute; (iii) filling out questionnaires for identifying psychological parameters for five minutes; and (iv) taking a rest to eliminate residual sensitivity for five minutes. The physiological parameters were measured in steps (i) and (ii), in which the measurement in step (i) was not an absolute, stable value but a certain level of stimulation given by the gray screen. In step (ii), six groups (cases) that can be consist of three ECD images were created, these groups were randomly ordered, and were displayed sequentially to the participants. The process from step (i) to step (iv) was repeated three times until the participant looked at all three images of the ECDs.

The experimental procedure is shown in Fig 1.

**Fig 1:** Experimental procedure performed in this study. The order of the stimulus conditions was varied to avoid order bias. The erosion control dam, heart rate, heart rate variability, semantic differential method, and profile of mood state were abbreviated to ECD, HR, HRV, SD, and POMS, respectively.

Visual stimulation was conducted using a 4K compatible high vision liquid crystal display device of 1240 mm width, 714 mm height, and 3840 × 2160 pixel resolution. The device displayed one of the following three images in full size: (i) an ECD featuring that the concrete wall surface with pattern of grooves engraved using formwork was exposed (concrete-exposed); (ii) an ECD featuring that the layers of stones with 0.5−1.0 m in diameter were horizontally attached on top of one another on the concrete wall surface (stone-attached); and (iii) an ECD featuring that the embalmed wood slats were horizontally attached on top of one another on the concrete wall surface (wood-attached) (Fig 2). All other elements that could interfere with the landscape perception, such as the ECD’s width and height, the surrounding vegetation cover, and stream water surface and discharge, were handled using Adobe Photoshop CS6 software (version 13).

**Fig 2:** The images of erosion control dams (ECDs) with three different exteriors. (a) Concrete-exposed ECD, (b) Stone-attached ECD, and (c) Wood-attached ECD.

### 3. Physiological indicators

HR and HRV, which are commonly used to quantify autonomic nervous activity, were measured using a wearable electrocardiogram sensing system (myBeat; Union Tool Co., Tokyo, Japan) [33]. The HRV was analyzed for the periods between two consecutive R waves (R–R intervals) in the electrocardiogram [34], and the power levels of low-frequency (LF; 0.04–0.15 Hz) and high-frequency (HF; 0.15–0.40 Hz) components derived from the HRV were calculated using the maximum-entropy method (Memcalc/Win, GMS, Tokyo, Japan) [35]. The HF parameter reflected parasympathetic nervous activity, which is activated during a physiologically relaxed state, and the LF/HF parameter reflected sympathetic nervous activity, which is activated during a state of stress and awareness [36].

### 4. Psychological indicators

#### 4.1. Semantic differential (SD) method

The SD method, a questionnaire that evaluates the impression of an object using adjectives that express human sensitivity [37], was used to assess the participants’ responses to the stimuli. The number of adjectives used in the SD method varies depending on the study’s purpose (e.g., [38–41]). Herein, we used six opposing adjective pairs, ‘natural–artificial’, ‘clean–dirty’, ‘friendly–unfriendly’, ‘calm–dynamic’, ‘peaceful–unpeaceful’, and ‘relaxed–anxious’, which can be felt intuitively from the exterior of an ECD. Of the two adjectives in each pair, the distinction between words with positive and negative meanings was determined by considering the fundamental conditions that an ECD should have as part of nature. A seven point Likert scale consisting of integers from –3 to +3 was applied, and a relatively higher Likert score for a given adjective pair meant that participants perceived positively.

#### 4.2. Profile of mood state (POMS)

The POMS is a well-established measure of psychological distress derived from factor analysis [42, 43]. We assessed participants’ temporary mood states for particular stimuli using the Korean POMS (K-POMS-B), which is a brief version of the POMS and is modified by Yeun and Shin-Park [44]. It consists of 30 items including questions, such as ‘tense’, ‘sad’, ‘angry’, ‘worn out’, ‘confused’, and ‘lively’. Each item is evaluated on a five point Likert scale consisting of integers from zero to four and is included in one of six theoretical mood factor subscales: tension–anxiety (T), depression (D), anger–hostility (A), fatigue (F), confusion (C), and vitality (V), so each subscale includes five items. However, in the case of ‘efficiency’, one of the five items corresponding to the confusion (C) subscale, the original rating values were reversed, i.e., 0–4, 1–3, 2–2, 3–1, and 4–0, to maintain a consistent meaning with the other items in the subscale [45].

The scores of the items corresponding to each subscale were summed from the questionnaire filled out by each participant, and the sum was substituted into the formula T+D+A+F+C–V to estimate the total mood disturbance (TMD) score for each participant.

### 5. Data analysis

Before the analyses, 2 of a total of 34 participants were excluded from the data analyses using HRV data because of errors in the HRV data collection. In addition, the HF and LF/HF parameters were transformed into their natural logarithmic values, ln(HF) and ln(LF/HF), respectively, to standardize the variances and improve normality [46]. The normality of the distributions was tested using the Kolmogorov–Smirnov test. The analyses of physiological parameters were performed using HR, ln(HF), and ln(LF/HF) as well as the changes (△HR, △ln(HF), and △ln(LF/HF)) from certain levels of stimulation values measured while viewing the images of the ECDs.

Repeated measures analysis of variance (ANOVA) was performed for the statistical analysis of physiological parameters, and the Friedman test was performed for the statistical analysis of psychological parameters. Post hoc comparisons using Bonferroni’s correction were performed for both physiological and psychological parameters. Furthermore, to estimate the effect sizes, we calculated eta-squared for the physiological indicators and Kendall’s coefficient of concordance for the psychological assessments.

All statistical analyses in this study were carried out with the statistical package SPSS, version 29.0 (IBM Corp., Armonk, NY, USA), and a *p* of < 0.05 indicated statistical significance for all tests. All values are expressed as means ± standard errors.

## Results

### 1. Changes in physiological indicators depending on the ECD images displaying three different exteriors

The mean value of participants’ HRs measured before and while viewing the images of the three ECDs ranged from approximately 73.40 bpm to 73.82 bpm and from 73.10 bpm to 74.38 bpm, respectively, and no significant difference was found between them (*p* > 0.05) (Fig 3A).

**Fig 3:** Comparison of (a) HR and (b) △HR between three ECDs (*n* = 34; *p < 0.05 using repeated measures analysis of variance (ANOVA) with Bonferroni’s correction). The values are expressed as means ± standard errors. The erosion control dam and heart rate are abbreviated to ECD and HR, respectively.

The △HR was slightly increased when viewing the images of the concrete-exposed ECD (0.98 ± 0.52 bpm) and the stone-attached ECD (0.31 ± 0.65 bpm), whereas it was slightly decreased when viewing the image of the wood-attached ECD (–0.71 ± 0.40 bpm) (Fig 3B). A significant difference was found only between the images of the concrete-exposed ECD and the wood-attached ECD (*p* < 0.05; η^2^ = 0.093).

The mean value of ln(HF)s extracted from the participants’ HRVs measured before and while viewing the images of the three ECDs ranged from 5.78 lnms^2^ to 5.81 lnms^2^ and from 5.82 lnms^2^ to 5.86 lnms^2^, respectively, and no significant difference was found between them, as with the HRs (*p* > 0.05) (Fig 4A). The △ln(HF) showed a relatively larger increase when viewing the image of the concrete-exposed ECD (0.08 ± 0.11 lnms^2^), followed by the wood-attached ECD (0.03 ± 0.09 lnms^2^), and the stone-attached ECD (0.02 ± 0.11 lnms^2^) (Fig 4B). However, all showed positive values regardless of the ECD image, and there was no significant difference (*p* > 0.05).

**Fig 4:** Comparison of (a) ln(HF) and (b) △ln(HF) between three ECDs (*n* = 32; no significant difference using repeated measures analysis of variance (ANOVA) with Bonferroni’s correction). The values are expressed as means ± standard errors. The erosion control dam and high-frequency power level are abbreviated to ECD and HF, respectively.

The mean value of ln(LF/HF)s extracted from the participants’ HRVs measured before and while viewing the images of the three ECDs ranged from 0.22 to 0.43 and from 0.13 to 0.25, respectively, and no significant difference was found between them, as with HR and ln(HF) (*p* > 0.05) (Fig 5A).

**Fig 5:** Comparison of (a) ln(LF/HF) and (b) △ln(LF/HF) between three ECDs (*n* = 32; no significant difference using repeated measures analysis of variance (ANOVA) with Bonferroni’s correction). The values are expressed as means ± standard errors. The erosion control dam and low and high-frequency power levels are abbreviated to ECD, LF, and HF, respectively.

The △ln(LF/HF) showed a slight increase when viewing the image of the concrete-exposed ECD (0.01 ± 0.15), whereas it decreased when viewing the images of the stone-attached ECD (–0.18 ± 0.16) and the wood-attached ECD (–0.16 ± 0.15) (Fig 5B). However, as with ln(HF), there was no significant difference between them (*p* > 0.05).

### 2. Changes in psychological indicators depending on the ECD images displaying three different exteriors

The results of the SD method show that participants perceived the concrete-exposed ECD (–1.26 ± 0.33 points) and the stone-attached ECD (–0.38 ± 0.38 points) artificially, while they perceived the wood-attached ECD (1.12 ± 0.32 points) naturally (*p* < 0.05; W = 0.369) (Fig 6A). However, it was confirmed that the participants showed clean, friendly, calm, peaceful, and relaxed perceptions of all the ECDs based on the statistical analysis results. Furthermore, there was no statistically significant difference between the ECDs with three different exteriors in these five questionnaire items used in the SD method (*p* > 0.05), even though their scores differed according to the ECD’s exterior type (Fig 6B–6F).

**Fig 6:** Comparison of SD method scores between three ECDs (*n* = 34; *p < 0.05 using Friedman test with Bonferroni’s correction). The scores are expressed as means ± standard errors. The erosion control dam is abbreviated as ECD.

The results of the K-POMS-B analysis statistically show that the participants did not express differences according to the ECD’s exterior for items corresponding to negative moods such as T, D, A, F, and C, although their values were somewhat different (Fig 7A–7E). On the other hand, for the items corresponding to V, a positive mood, a difference according to the ECD’s exterior was shown, that is, participants’ scores for the concrete-exposed ECD (3.29 ± 0.69 points) or the stone-attached ECD (3.38 ± 0.67 points) were significantly different from that for the wood-attached ECD (5.59 ± 0.79 points) (*p* < 0.05; W = 0.214) (Fig 7F).

**Fig 7:** Comparison of six theoretical mood factors and TMD scores estimated using K-POMS-B between three ECDs (*n* = 34; *p < 0.05 using Friedman test with Bonferroni’s correction). The scores are expressed as means ± standard errors. The erosion control dam, six theoretical mood factors (tension–anxiety, depression, anger–hostility, fatigue, confusion, and vigor), and total mood disturbance are abbreviated as ECD, T, D, A, F, C, V, and TMD, respectively.

The participants’ TMD scores, estimated by substituting all subscales’ scores into the formula T+D+A+F+C–V, showed a relatively larger increase for the concrete-exposed ECD (5.65 ± 1.57 points), followed by the stone-attached ECD (4.74 ± 1.54 points), and the wood-attached ECD (1.68 ± 1.50 points). Significant differences in the TMD scores were found only between the concrete-exposed ECD and the wood-attached ECD (*p* < 0.05; W = 0.213) (Fig 7G).

## Discussion

An ECD is an infrastructure for reducing or preventing sedimentary disasters that can be caused by geomorphic disturbances in stream water zone. Above all, it should have physical stability against external forces. Mizuyama and Matsumura [47] and Chun [11] presented four stability conditions that an ECD should satisfy structurally: (i) stability against falling; (iii) stability against sliding; (iii) stability against dam body destruction; and (iv) stability against the bearing capacity of the foundation ground. Although an ECD should be designed and constructed creatively in consideration of the on-site and surrounding conditions (e.g., stream water peak discharge, the plane and cross sectional profiles of stream, stream bed materials, etc.), it is reasonable to assume that the four stability conditions can be secured if the guidelines for the design and construction methods are thoroughly followed since an ECD does not contain many types of construction materials, and many of them are standardized. This study, therefore, intended to discuss the necessity and methodology of evaluating the natural landscape created by the artificial installation of an ECD infrastructure, which already has sufficient stability against sedimentary disasters in stream water zone.

In this study, we examined participants’ physiological and psychological responses while they viewed images of ECDs of three different exterior types (i.e., concrete-exposed, stone-attached, and wood-attached). The experimental process was similar to that of a previous study by Annerstedt et al. [48], who determined the effect of participants’ stress recovery when they did and did not view a forest landscape after using the Trier Social Stress Test (TSST) to cause stress using the physiological indicators HR and HRV. It was also similar to Park et al.’s study [49], which examined the relationship between psychological responses using the psychological indicators in the SD method and POMS and the physical environment after sitting–viewing and walking in each target site in the forest and urban environments. However, this study is original in that it quantified only the effects of the exterior of an ECD. Moreover, it is different from their research because we did not use extremely conflicting experimental conditions, such as the presence or absence of forests or cities. Furthermore, this study drew complementary conclusions using both physiological and psychological indicators like Kim and Song [33], Kim et al. [50], and Song et al. [51].

No significant difference was found between the participants’ HRs measured before and while viewing the images of the three ECDs finished with different exterior materials, and the △HR did not exceed ± 1.0 bpm in all cases (Fig 3). Jo et al. [52] compared the changes in participants’ HRs (△HRs) between viewing images with a broad scale mountain landscape of the autumn foliage season and an urban landscape including skyscrapers and reported no significant difference between the two images. However, the △HR decreased by approximately 0.64 ± 0.50 bpm when viewing the mountain image, which is similar to our results for the wood-attached ECD (0.71 ± 0.40 bpm). This means that the △HR shown for the wood-attached ECD was not a very large value. However, a significant difference was detected in the △HRs between the concrete-exposed ECD and the wood-attached ECD (Fig 3B). This result clearly shows that the participants responded consistently to each stimulus given by concrete (artificial material) and wood (natural material), and agrees with the previous study by Kim [53], who conducted a preference evaluation of 12 road paving materials and reported that while concrete gave an artificial feeling, wood was perceived as natural. In addition, Song et al. [54], who compared the HRs measured with participants walking–viewing the scenery of an urban park and city area (86.7 bpm and 90.3 bpm), and Song et al. [55], who compared the HRs measured with participants sitting–viewing the scenery of a forest area and an urban area (75.3 bpm and 80.6 bpm), also reported that significant differences between the two opposing stimuli of natural vs. artificial or green vs. gray. This trend is similar to the findings of the present study.

The trend in these HR indicators was similar to that in the HRV indicators, that is, the ln(HF), an indicator of parasympathetic nerve activity, and the ln(LF/HF), an indicator of sympathetic nerve activity, showed no significant differences due to the differences in exteriors of the ECDs as well as the observation of the ECD images. Moreover, the △ln(HF) and △ln(LF/HF) increased up to 0.08 lnms^2^ (for the construct-exposed ECD) and decreased up to 0.18 (for the stone-attached ECD), respectively (Fig 4). This can be interpreted as a fairly insignificant change. Song et al. [55] found that the △ln(HF) and △ln(LF/HF) significantly increased and decreased when viewing real forests and urban landscapes, respectively. These results indicate that viewing forest landscapes induces physiological relaxation by increasing parasympathetic nerve activity and suppressing sympathetic nerve activity. There was no statistically significant difference in this study, but the trends were consistent with these studies. Song et al. [40] analyzed the △ln(HF) and △ln(LF/HF) caused by forest derived visual, auditory, and visual and auditory combined stimulation, and reported that the △ln(HF) and △ln(LF/HF) for forest derived visual stimulation exhibited insignificant levels (△ln(HF): approximately 0.2 lnms^2^; △ln(LF/HF): approximately 0.21). Although they only dealt with healthy women in their early 20s, their findings indirectly show that the differences in the ln(HF) and ln(LF/HF) and increases or decreases in the △ln(HF) and △ln(LF/HF) identified in this study were not at remarkable levels considering the results did not significantly differ depending on the participant’s gender, as in several previous studies (e.g., [56, 57]), which evaluated the effects of landscape images via displays of virtual reality.

As additional and supplementary indicators to physiological responses described above, the psychological parameters also did not significantly deviate from the previous results and discussion. The results of the SD method show that all participants responded positively regardless of the exterior of the ECDs (Fig 6B–6F). The studies by Park et al. [49], Tsunetsugu et al. [58], Joung et al. [59], Song et al. [30], Song et al. [55], and so on reported that forests give clean, friendly, calm, peaceful, and relaxed impressions compared with objects other than forests. Although their studies are different in that they targeted relatively extremely opposing conditions (such as the presence vs. absence of forests, or cities vs. forests) compared with this study, the results of the present study show that an ECD is recognized as a part of the forest prior to recognition of its exterior. There was, however, a significant difference in the scales of artificial vs. natural, which indicates the intuitive effect of the exterior material (Fig 6A). This can be explained as an extension of the discussion about the results of the △HR analysis in Kim’s study [53] and this study.

Regarding the K-POMS-B results, there were no significant differences in participants’ scores indicating the negative mood categories of T, D, A, F, and C according to the exteriors of the ECDs, ranging from approximately 0.26 to 4.79 out of 20 points (Fig 7A–7E). This can be interpreted as them receiving a less negative perception than the urban environment, regardless of the exterior material of the ECD. Jo et al. [60] compared the physiological and psychological responses to viewing two images displaying a beautiful waterfall and a large asphalt road across high rise buildings. The score ranges of all negative subscales with the POMS in their study were distributed from approximately 0.11 to 1.78 points when viewing the image of a waterfall and from approximately 0.74 to 4.89 points when viewing the image of an asphalt road. The scores in this study were distributed in the interval between them. In addition, the study by Song et al. [55], which showed landscapes of a forest area and an urban area to participants and obtained negative subscale scores of approximately 0.1 to 4.0 points and 0.6 to 4.6 points, respectively, also included the score range in this study. However, the score of the V subscale, a positive category, was lower than that (approximately 7.07 points) of the waterfall image presented by Jo et al. [60] and was higher than that (approximately 2.2 points) of the real forest landscape presented by Song et al. [55], indicating that the participants felt relatively positive perceptions. It was found that the natural materials induced a relatively more positive perception, as the wood-attached ECD showed a significant difference compared with the concrete-exposed ECD and the stone-attached ECD. It is judged that this difference contributed to the lowest TMD score of the wood-attached ECD. However, considering the TMD scores (waterfall: −2.15 ± 1.35 vs. urban: 11.26 ± 2.39, as presented by Jo et al. [60]; forest area: 4.8 ± 0.6 vs. urban area: 11.9 ± 1.1, as presented by Song et al. [55]) in these previous studies, the TMD scores of the concrete-exposed ECD or the stone-attached ECD in this study were much closer to that of the forest area than that of the urban area.

As mentioned above, the participants’ physiological and psychological responses to the exteriors of the ECDs were found to be overall positive. This may be because the three images used in the experiment of this study contained a nature-positive landscape with vegetation fully covered and stream water flowing around the ECDs. Lee et al. [18] evaluated the importance of landscape factors including elements of the ECD, such as the material and size, as well as elements around the ECD, such as the extent of vegetation cover and presence of stream water. They reported that the extent of vegetation cover and presence of stream water around the ECD were evaluated as relatively important factors. Preserving the landscape elements of an ECD is important; however, it may be even more important to keep the landscape surrounding the ECD with a nature-positive condition. To conclude, the design and construction of an ECD should be prioritized to secure stability against potential sedimentary disasters in stream water by satisfying the four stability conditions before selecting the exterior materials considering the landscape. However, as an ECD that is constructed in an urban living area with a highly concentrated population is easily exposed to local residents, it is necessary to maintain the vegetated and stream water flowing surroundings of the ECD, and apply natural materials to its design and construction so that physiological and psychological stabilities can be maximized within the range allowed by the budget.

## Conclusions

In everyday life, people visit urban green spaces surrounding a living area to enjoy nature away from artificial structures. However, artificial structures of various forms and functions can be seen even in green spaces. In countries with vulnerability to sedimentary disasters such as South Korea, Japan, China, Italy, Spain, and Austria, ECDs, which are a gray infrastructure for reducing risk due to sedimentary disasters in stream water zone, can often be seen within green spaces, which are the green infrastructure surrounding an urban area [61–65]. Our findings show that people do not physiologically and psychologically perceive ECDs negatively, although the wood-attached ECD induced a slightly more positive perception compared to the concrete-exposed ECD and the stone-attached ECD in this study. Therefore, securing stability against potential sedimentary disasters should be the top priority for the design and/or construction of an ECD, and after satisfying this prerequisite, it would be desirable to use nature-positive materials such as wood as the landscape elements of an ECD.

As this is a pioneering study that deviates from the existing landscape evaluation technique for ECDs, some parts need to be supplemented in future studies. First, the present study primarily aimed to examine the physiological changes associated with the evaluation of the landscape created by ECD, and for this purpose, the sample size was calculated by assuming the one-way ANOVA for analyzing physiological indicators. This may lead to the calculation of insufficient sample size to accurately estimate the effect size of psychological assessments. Therefore, follow-up studies dealing with larger sample size with various age groups should be conducted, and if possible, the process of organizing and analyzing data should be able to secure higher reliability and transparency through pre-registration. Second, this study was conducted based on a somewhat balanced gender composition (i.e., 19 males and 15 females). However, since gender composition can be critical confounding variable in the field environmental physiology and psychology, studies including gender composition as one of the variables should be followed in the future. Third, the ECD landscape should be evaluated based on the influence of the stimulation of the five senses in an actual forest, in addition to considering the effect of visual stimulation in a space where all conditions are controlled, such as in this study. This should be carried out while considering the significant influences of the type of stimulus as well as individual preferences, interests, and values. Finally, since an ECD can be distinguished not only by its exterior materials but also by its structural type (open type vs. closed type), follow up landscape evaluations for various types of ECDs should be carried out. These future studies are essential to secure the objectivity of the evaluations of not only the landscape created by ECDs but also the function of protecting the human living sphere from sedimentary disasters and further enabling a healthy forest and stream ecosystems to be sustainable.

## Supporting information

S1 Table (XLSX)

S2 Table (XLSX)

S3 Table (XLSX)

S4 Table (XLSX)

S5 Table (XLSX)

S6 Table (XLSX)
